This article has been retracted.

# Analysis of the Stage Performance Effect of Environmental Protection Music and Dance Drama Based on Artificial Intelligence Technology

**DOI:** 10.1155/2022/2891993

**Published:** 2022-09-19

**Authors:** Li Zeng

**Affiliations:** Jiangxi Science & Technology Normal University, Nanchang 330000, China

## Abstract

There are a lot of environmental protection musicals and dances in public entertainment life to support the concept of environmental protection and to entice people to support the cause of environmental protection. As we all know, in a musical performance, the distance between the audience and the actors, the design of the stage environment, the training of the actors, the costumes of the actors, the makeup of the actors, and the musical accompaniment will all have more or less influence on the stage performance effects. In order to make environmental protection music and dance dramas profoundly meaningful to social production and human activities, it is especially important to analyze the stage performance of such music and dance dramas. The analysis of stage performance effects is not only beneficial to making the ideas spread by the music and dance drama penetrate into people's hearts but can also provide guiding suggestions for the production of music and dance drama. Therefore, this paper proposes a linear regression algorithm based on artificial intelligence to deeply explore and analyze the influence of the above six factors on the stage performance effects of environmental protection music and dance drama. In our method, first we preprocess the data collected by classification to remove the odd values from the data so that the various types of data conform to a normal distribution. Secondly, we obtained linear fit plots of the six factors with the stage performance effect scores by using a linear regression algorithm to deeply analyze the correlation between various types of data and the stage performance effect scores. Finally, through numerical calculations, we found that the distance between the audience and the actors, the training of the actors, and the musical accompaniment have a greater influence on the performance effect of the musical cabaret in the environmental protection category. Meanwhile, the costumes of the actors, the makeup of the actors, and the design of the stage environment have less influence on the performance effect of the musical cabaret. Therefore, in the production and performance of environmental protection music and dance dramas, producers and performers should pay more attention to the distance between the audience and the actors, the design of musical accompaniment, and the training of actors. To sum up, this paper has made a scientific, detailed, and reasonable analysis of the performance effect of environmental protection music and dance dramas on stage, contributing to the dissemination of environmental protection ideas.

## 1. Introduction

As the Earth's environment continues to deteriorate, humans will face many deadly threats. For example, the continued rise in temperature in Antarctica will cause the sea level to rise. The melting of permafrost will release gases containing unknown viruses. The African continent's plate split [1]. Large amounts of toxic plastic particles in the Arctic snow emerge. These issues compel us to protect and improve the Earth's environment, which is the only way to reduce unpredictable and deadly threats. However, protecting the environment is not something that can be done by just one person [2]. Although people's awareness of environmental protection has increased, the situation of environmental pollution and resource waste is still serious, and there are many people who still do not take action to protect the environment. Therefore, in order to spread the idea of environmental protection and call for people to participate in activities to protect the environment, there are many environmental protection music and dance dramas appearing in the entertainment lives of the public [3, 4]. The most direct and easily felt consequence of environmental pollution is that it degrades the quality of the human environment and affects the quality of human life, physical health, and productive activities.

People began to consider their own authoritarian attitudes about nature during the 1980s as they became aware of how dramatically the environment was changing. French dancers came to value the use of dance to explore the relationship between natural space and human beings [5, 6]. For example, the French modern dance choreographer Kibova, who created *Dance for Four* and *Movement* in 1980, has a creative idea according to the promotion of environmental protection. Daniel's *Waterproof* was performed in a real swimming pool, where the weightlessness and floating of people in the water were expressed by the dance. The relationships between people and water, people and people, and people and their surroundings are all presented in the water by the dance. This dance brings to light that human behavior in a water environment is quite different from that on land [7]. With the deterioration of the environment, environmental music and dance theater have been developing. French choreographers have often introduced film, television, and theater to dance, making environmental music and dance theater a truly comprehensive theater art. Currently, environmental protection music and dance theater are contemporary art forms of concern in many developed countries, where dancers improvise through the human body to express their perception of the environment, architecture, nature, or urban space. At the same time, they use pictures and images to record in time, recreate in the record, and dig deeper into the complex and subtle relationship between people, the urban environment, and architecture. Let the viewer feel the strong visual impact and look at our lives and living environment with new eyes to discover the essence of life [8, 9].

An excellent musical song and dance drama not only give the audience a good experience but also promote the dissemination of the ideas preached by that musical and dance drama and even promote the development of the musical song and dance drama. The good or bad stage performance of the musical song and dance drama determines the success or failure of the musical song and dance drama. In particular, environmental protection music and dance drama should have good stage performance, which will not only cause people to realize the harm of environmental degradation but also call on people to consciously restrain their own behavior and join the trend of environmental protection [10]. Therefore, the stage performance of environmental protection music and dance drama is an issue that writers and producers should think about in advance. There are many factors that affect the stage performance of environmental protection music and dance drama, including the distance between the audience and the actors, the design of the stage environment, the training of the actors, the costumes of the actors, the makeup of the actors, and the musical accompaniment. Here, we will explain how these factors affect the stage performance of environmental protection music and dance dramas in the following [11].

The audience is the appreciator, and without the audience, there is no performance. The audience is the core of the performance; the actor brings life and soul to the performance; and the audience receives the artistic beauty and emotion brought by the performance [12]. As an audience, there is a certain spatial distance from the stage from which it is impossible to see just one actor and observe every detailed action. As a standard outsider, they are often more able to see where the problems with the performance lie. In the musical cabaret, they can even see which actor made a small gesture. An excellent musical cabaret is precisely through the details to send strong emotional signals to the audience, causing the audience to resonate. When an audience watches a performance, they are bound to react emotionally to the performance on stage. The audience will directly express through their emotions how good or bad the musical cabaret is. Such emotions generated by the audience will not only affect the emotions of other theatergoers but also the emotions of the actors on stage [13].

Stage environment design is the most important part of stage visual artists' attention, which plays an important role in the expression and audience's understanding of musical cabaret. In stage environment design, the environment and the size of the venue in which the musical cabaret is viewed will have an impact on the performance. The mood conveyed by the use of space structure will draw the attention of the audience and continue to play an important role. During the performance, different changes in the mood of the space will also bring new visual experiences to the audience. With the development of science and technology, new technologies are slowly dipping into music, song, and dance dramas [14, 15]. Transforming these new technical languages into stage environment design will transfer new energy to environmental protection music, song, and dance dramas and will promote the spread and development of environmental protection music, song, and dance dramas.

The training of actors is an important way to develop the performance abilities of music and dance theater actors. The daily training is very rich and diverse, including both professional training in performance and training in psychological adjustment ability. Specifically, the daily training includes line ability, cultural training, movement ability, mental regulation ability, logical thinking and analysis ability, and other aspects of training [16]. For musical cabaret performers, daily training is the most arduous and boring. Daily training not only requires actors to have tenacity and tough character but also requires instructors to have scientific training methods to constantly help actors overcome inertia while effectively improving the level of training and respecting the laws of art, so that actors can gain improved acting ability in the shortest possible time.

For performers, there is more to performance costumes than simply a piece of clothing. The performance costume is the interpretation of the soul of the entire stage art and serves as an important prop to shape the external image of the character. A unique and effective costume can make the performers shine [17]. Specifically, the choice of costumes for the performers of environmental protection musicals and dances will influence the artistic image of the performers and the style of their performance. For example, children's performance clothes are more colorful, highlighting the lively and lovely children; the performance clothes of the elderly are relatively single color, highlighting the maturity and stability of the elderly.

Actor makeup is an important part of the art of the stage, helping to express the character and enhance the artistic expression of the stage [18]. Stage makeup is different from daily makeup; it needs to be closely matched with stage lighting and actors' costumes in terms of color and tone to achieve the best stage effect. Successful stage makeup contributes to an actor's expressiveness and can add color to the stage effect. A good makeup artist should not only focus on improving his or her skills and artistic training but also on cooperating with lighting artists, costumers, etc., using lighting and costumes to assist in the display of makeup effects. The makeup of the actor is a visual embellishment, which directly affects the appreciation value of the stage performance. The types of stage performances and the various characters are beautified with cosmetic tools in order to combine them with the content of the story.

Stage performance in the musical accompaniment can be accompanied by the performance of the content of continuous enrichment and, then in the process of interpretation, will naturally give the whole performance a more complete expression. The musical accompaniment is an essential part of the stage performance, and the musical accompaniment has more expressive power in the stage performance [19]. Music itself has the role and power to influence people's thoughts and feelings, and the flow of music melody has a direct impact on the movement of the human body and people's emotional changes. Harmonious and beautiful musical accompaniment can drive the passion of performers. A successful and influential musical cabaret requires a corresponding musical accompaniment to make it more complete. The aural art infection can stimulate the performance subject to perform more richly, encourage him to maintain a good state of mind for the whole performance at all times, and allow him to better grasp the feeling of performance and the expression of emotion in the process of interpretation. In turn, the whole stage performance effect has rich infectious power and enjoyable performance art.

Only when an actor has good line skills can he or she smoothly convey information to the audience in the process of performance, better portray the character, and promote the development of the plot. The actor's cultural cultivation directly determines the actor's acting ability and artistic achievement. Without good cultural cultivation, it is impossible for an actor to deeply understand the script, life, and role and to use acting skills to better portray the character on stage. With good movement ability, the theater actor will be able to better master the rhythm in the process of performance, to be relaxed and natural and steady, to better use body language to convey information, and to make the character's image more fleshed out [20]. In the course of a live performance, there are likely to be some temporary and sudden situations, including microphone loss, lighting failure, and audience reaction. All these sudden events and factors will have some impact on the actor's live performance. The most successful group of supervised learning models in machine learning is linear regression models. Despite being straightforward, they are crucial and serve as the foundation for many intricate models.

In order to thoroughly study and analyze the impact of the aforementioned six parameters on the stage performance effect of environmental protection class music and dance drama, we present a linear regression algorithm based on artificial intelligence in this work. In this approach, the data gathered through classification is first preprocessed to weed out any outliers and guarantee that the different categories of data are distributed regularly. Second, we thoroughly examined the relationship between various types of data and stage performance effect scores after obtaining linear fit plots of six components and stage performance effect scores using a linear regression technique. Finally, we discovered by numerical analysis that the audience-actor distance, actor training, and musical accompaniment have a stronger impact on the performance effect of musical cabaret in the field of environmental protection.

## 2. Related Works

Yan and Wang [18] compared the technical systems of outdoor live performance stages and indoor theater stages and proposed a unique stage effects presentation technology for outdoor live performance stages. Ardizzi et al. [21] conducted a study looking at the physiological responses of the audience and showed the expected increase in synchrony among those belonging to the same quartet during the viewing of the performance and during breaks. In addition, participants' cardiac synchrony was found to be associated with convergence in the audience's explicit emotional evaluation of the performance they were watching. These findings suggest that the mere copresence of others is sufficient for cardiac synchrony to occur spontaneously and that it increases in response to a shared and consistent explicit emotional experience. bin Paharul Rozi and Amirrul [22] used temu bual and pemerhatian methods and focused on the costumes of traditional plays in Pinan Island, identifying the understanding and function of costume elements in the costume components of each play. Their results show that the current costume variations have been concretized because the public is more attracted to them than to the actors' costumes.

Rahman et al. [23] examined the importance of musical theater, the definition of musical theater, the classification of song types and dramatic themes of performances, the impact of musical theater on students' development, and the advantages and disadvantages included in musical theater performances. Also, they described the important results of various previous studies on musical theater performances to increase students' motivation to study literature. Billeri [24] presented the first systematic analysis of the musical and external characteristics of the genre as popular theater and shows the process by which traditional forms were adapted to new audiences and performance environments, creating new forms of theater and dance. At the same time, they provide a general description of the origins of classical dance theater, costumes, characters, storylines, and ensembles related to performances of the last century. Oladipo and Akhigbe [25] focused on the design and implementation of the Performing Arts Enhanced Three Stage Instructional Model (PAEIM), which incorporates drama, dance, and music. Their results suggest that PAEIM is an effective model of performing arts instruction that greatly enhances conceptual understanding of actor training and influences students' self-determination and intrinsic motivation. It also showed that PAEIM improved the effectiveness of actors' stage presence when performing.

## 3. Modeling Methods

### 3.1. Linear Regression

Linear regression models are the most effective class of supervised learning models in machine learning. Although simple, they are the basis of many complex models and are very important [26, 27]. Linear regression deals with a class of problems where given a set of input samples and a target value corresponding to each sample, it is necessary to learn the relationship between the target value and the input value as a function of a certain loss criterion [28]. In this way, when a new sample arrives, it is possible to predict what its corresponding target value will be. Linear regression is the prediction of new data based on existing data, that is, the ability to describe the relationship between data more precisely with a straight line, so that when new data appears, a simple value can be predicted.  Figure 1 shows a flow chart of how the linear regression algorithm works.

The model of linear regression is shaped as

(1) $$\begin{array}{c} h\left(x\right)=w_{1}x_{1}+w_{2}x_{2}+w_{3}x_{3}+\cdots +w_{n}x_{n}+b, \end{array}$$

where *w* is the weight function, *b* is the deviation function, and *x* is the input variable.

The model from linear regression is not necessarily a straight line, but a straight line in a plane when there is only one variable [29, 30]. When there are two variables, the model is a plane in space. When there are more variables, the model will be higher dimensional.

Linear regression models have good interpretability and can be used to see directly from the weights *W* how much each feature affects the results. Linear regression is suitable for data sets where there is a linear relationship between *x* and *y*. A computer-aided scatter plot can be drawn to see if there is a linear relationship [31, 32]. We try to fit the data using a straight line so that the sum of the distances from all points to the line is minimized.

In fact, the sum of squared residuals, which is the distance from a point to a line parallel to the *y*-axis without using the vertical distance, is usually used in linear regression, and the sum of squared residuals divided by the sample size *n* is the mean squared error. The mean squared error is used as the loss function of the linear regression model [33]. Minimizing the sum of the distances from all points to the line minimizes the mean squared error, and this method is called least squares.

The loss function equation can be expressed as

(2) $$\begin{array}{c} J=\frac{1}{n}\overset{n}{\underset{i=1}{\sum }}{\left(y_{i}-h\left(x_{i}\right)\right)}^{2}. \end{array}$$

On the basis of equation (1), the final equations for *w* and *b* are obtained by solving the following:

(3) $$\begin{array}{c} w=\frac{\sum_{i=1}^{n}\left(\left(x_{i}-\bar{x}\right)\left(y_{i}-\bar{y}\right)\right)}{\sum_{i=1}^{n}{\left(x_{i}-\bar{x}\right)}^{2}}, \end{array}$$

(4) $$\begin{array}{c} b=\bar{y}-w\bar{x}. \end{array}$$

By analyzing the problem, determining the loss function or utility function of the problem and obtaining a model for machine learning by optimizing the loss function or utility function, this is the general set of parametric learning algorithms [34, 35].

The following is a brief description of the data processing process. Suppose the input data set *D* has *n* samples and *d* features; then,

(5) $$\begin{array}{c} D=\left(\left(x^{1},y_{1}\right),\left(x^{2},y_{2}\right),\cdots ,\left(x^{n},y_{n}\right)\right), \end{array}$$

where the *i*-th sample is denoted as

(6) $$\begin{array}{c} \left(x^{i},y_{i}\right)=\left(x_{1}^{i},x_{2}^{i},\cdots ,x_{d}^{i},y_{i}\right). \end{array}$$

The linear model makes predictions by building linear combinations [36]. Our assumption function is

(7) $$\begin{array}{c} h_{\theta }\left(x_{1},x_{2},\cdots ,x_{d}\right)=\theta_{0}+\theta_{1}x_{1}+\theta_{2}x_{2}+\cdots +\theta_{d}x_{d}, \end{array}$$

where *θ*_0_, *θ*_1_, ⋯, *θ*_*d*_ are the model parameter.

Let *x*_0_ = 1, *x*^*i*^ = (*x*_1_^*i*^, *x*_2_^*i*^, ⋯, *x*_*d*_^*i*^), be a row vector, so that we get

(8) $$\begin{array}{c} X={\left[\begin{array}{c} x^{0}\\ x^{1}\\ \vdots \\ x^{n} \end{array}\right]}_{n\times d},\theta ={\left[\begin{array}{c} \theta_{0}\\ \theta_{1}\\ \vdots \\ \theta_{d} \end{array}\right]}_{d\times 1},Y={\left[\begin{array}{c} y_{1}\\ y_{2}\\ \vdots \\ y_{n} \end{array}\right]}_{n\times 1}, \end{array}$$

where *X* is an *n* × *d* dimensional matrix and *θ* is a *d* × 1 dimensional vector; then, assume that the function (7) can be expressed as

(9) $$\begin{array}{c} h_{\theta }\left(X\right)=X_{\theta }. \end{array}$$

The loss function is the mean square error, which can be expressed as

(10) $$\begin{array}{c} J\left(\theta \right)=\frac{1}{2}{\left(X_{\theta }-Y\right)}^{T}\left(X_{\theta }-Y\right). \end{array}$$

The least squares method of solving for the parameters and the derivative of the loss function *J*(*θ*) with respect to *θ* can be obtained:

(11) $$\begin{array}{c} \nabla J\left(\theta \right)=2X^{T}\left(X_{\theta }-Y\right). \end{array}$$

Let ∇*J*(*θ*) = 0; we obtain

(12) $$\begin{array}{c} \theta ={\left(X^{T}X\right)}^{-1}X^{T}Y. \end{array}$$

### 3.2. Analysis of the Effect of Music Performance in Environmental Protection Themed Musical Cabaret Based on Linear Regression

Linear regression algorithm is an advanced correlation analysis method in artificial intelligence algorithm, which contains many important ideas in machine learning and has more advantages. For example, the idea is simple, easy to implement, rapid to model, and effective for small data volumes and simple relationships [37, 38]. At the same time, the linear regression algorithm is the basis for many powerful nonlinear models, and its results are well interpretable, which facilitates decision analysis. However, linear regression algorithms also have some disadvantages that are difficult to overcome. For example, linear regression algorithms are difficult to model for nonlinear data or polynomial regression with correlation between data features, and at the same time, it is difficult to represent highly complex data well [39, 40].

After analyzing the audience's rating data on the distance between the actors and the audience, the design of the stage environment, the training of the actors, the costumes of the actors, the makeup of the actors, and the musical accompaniment, we found that these data and the stage effect rating data in general have the characteristics of linearity, small amount of data, and simple data relationship. Therefore, these data sets have an innate fit with the linear regression algorithm. However, through the normal distribution test, we found that a small portion of these data did not conform to the normal distribution. Thus, we preprocessed this data to remove the odd values from them.  Figure 2 shows the preprocessing as well as the analysis of the correlation between the six influencing factors mentioned above and the stage performance score using a linear regression algorithm.

## 4. Discussion and Analysis of Results

The data in this paper uses the evaluation scores of a concert site audience on different indicators to test the validity of the relevant indicators, where the data size is 100,000 items, and the data content includes quantitative scores of the stage performance effect, the distance between the audience and the actors, the training of the actors, the musical accompaniment, the costumes of the actors, and the design of the actors' makeup environment. To enhance the credibility of the article, we give the characteristic values of the collected data in Table 1.

Figure 3 shows the fitting effect of stage performance effect and audience-actor distance. The rating of actor distance largely fits with the rating of stage performance effect, with a fit of 98.6%. It shows that the actor's distance has a greater connection to the stage performance effect rating. As an audience, there is a certain spatial distance from the stage; it is impossible to see just one actor and observe every detailed action. Therefore, audience seating arrangement is crucial.

Figure 4 shows the fit between the stage performance effect and actor training, where each audience member's rating of actor training is relatively uniform. It shows that the ratings of actor training largely fit with the ratings of stage performance effect, with a fit of 97.5%. It indicates that the actor's distance has a greater connection to the stage performance effect rating. Therefore, we have to avoid some temporary and sudden conditions during the proscenium performance, including microphone loss, lighting failure, and audience proscenium reaction. These sudden events and factors can cause some impact on the actors' live performance.

Figure 5 shows the fit between the stage performance and the musical accompaniment, with each audience member rating the musical accompaniment more evenly. It shows that the rating of musical accompaniment is largely fitted with the rating of stage performance, with a fit of 95.2%. It indicates that the training of actors has a greater connection with the rating of stage performance effect. It can be seen that the musical accompaniment can enrich the performance continuously and make the musical cabaret more infectious.

Figure 6 shows the fitting effect of stage performance effect and actor's costume; each audience's rating of actor's costume is more scattered. It indicates that the ratings of the actors' costumes are poorly fitted to the ratings of the stage performance effect, with a fit of 75.9%. It indicates that the actor's costume has a small connection to the stage performance effect rating. Therefore, the diversity of audience aesthetics leads to a small correlation between actor's costumes and the performance effect evaluation of musical cabaret.

Figure 7 shows the fitting effect of stage performance effect and actor's makeup; each audience's rating of actor's makeup is more scattered. It indicates that the rating of actor's makeup has a poor fit with the rating of stage performance effect, with a fit of 69.7%. It means that the actor's makeup has a small association with the stage performance rating. The reason for this may be that the audience does not pay much attention to the actors' makeup.

Figure 8 shows the fitting effect of stage performance effect and environmental design; the rating of environmental design by each audience is more scattered. It indicates that the rating of environmental design is poorly fitted to the rating of stage performance, with a fit of 65.8%. It indicates that the design of the environment has a small connection to the rating of stage performance effect. Therefore, the design of the stage environment has less relevance to the performance and audience understanding of the musical cabaret.

## 5. Conclusions

Environmental protection music and dance drama are now an important way to promote environmental protection and an important art form to promote the spirit of environmental protection. A good stage performance is not only beneficial to making the ideas spread by the musical cabaret deeply rooted in people's hearts but can also provide guiding suggestions for the production of other types of musical cabarets. For the music and dance drama of environmental protection, we used the linear regression algorithm in artificial intelligence technology to analyze the six key factors affecting the stage performance effect. We used 100,000 quantitative ratings from a live concert audience for our experiments, where the ratings included audience-actor distance, actor training, musical accompaniment, actor costumes, actor makeup, and design of the environment. The experimental results revealed a 98.6%, 97.5%, and 95.2% correlation between the stage performance effect score and the distance between the audience and the actors, the actors' training, and the musical accompaniment, indicating that these three factors had a greater influence on the stage performance effect of environmental protection class music and dance drama. On the other hand, the correlations between the stage performance effect scores and actors' costumes, actors' makeup, and environmental design were 75.9%, 69.7%, and 65.8%, respectively, which indicated that these three factors had less influence on the stage performance effect of environmental protection music and dance dramas. To sum up, the proposed method has scientifically and rationally analyzed the relevance of factors influencing the stage performance of environmental protection music and dance dramas. At the same time, the results of this paper also provide important suggestions for the production of environmental protection music and dance dramas. Therefore, in the production and performance of environmental protection music and dance dramas, producers and performers should pay more attention to the distance between the audience and the actors, the design of musical accompaniment, and the training of actors.

## Figures and Tables

**Figure 1:** Flow chart of linear regression algorithm execution.

**Figure 2:** Preprocessing process and linear regression algorithm model diagram.

**Figure 3:** Fitting effect of stage performance effect and audience-actor distance.

**Figure 4:** Fitting effect of stage performance effect and actor training.

**Figure 5:** Fitting effect of stage performance effect and musical accompaniment.

**Figure 6:** Fitting effect of stage performance effect and actor's costume.

**Figure 7:** Fitting effect of stage performance effect and actor's makeup.

**Figure 8:** Fitting effect of stage performance effect and environment design.

**Table 1:** Scoring metrics for selected data.

Indicators	Audience 1 scoring	Audience 2 scoring	Audience 3 scoring
Stage performance effects	95	89	94
The distance between the audience and the actors	94	88	97
Training of actors	96	94	91
Musical accompaniment	90	73	88
Costumes for actors	88	65	77
Makeup for actors	75	79	86
Design of the environment	86	81	72

## Data Availability

The labeled data set used to support the findings of this study is available from the corresponding author upon request.
